This article has been retracted.

# LINC00152 down-regulated *miR-193a-3p* to enhance MCL1 expression and promote gastric cancer cells proliferation

**DOI:** 10.1042/BSR20171607

**Published:** 2018-05-08

**Authors:** Yong Huang, Hui Luo, Fang Li, Yun’e Yang, Guangsheng Ou, Xiaolong Ye, Nianchu Li

**Affiliations:** 1 Department of Gastrointestinal Surgery, Third Affiliated Hospital of Sun Yat-Sen University, Guangzhou 510630, Guangdong, China; 2 Anesthesia Surgery Center, Lingnan Hospital, Third Affiliated Hospital of Sun Yat-Sen University, Guangzhou 51000, Guangdong, China; 3 Supply Room, Lingnan Hospital, Third Affiliated Hospital of Sun Yat-Sen University, Guangzhou 51000, Guangdong, China; 4 Department of Hepatobiliary Surgery, Nanning Second People’s Hospital, Nanning 530031, Guangxi, China

**Keywords:** gastric cancer, LINC00152, miR-193a-3p, MCL1

## Abstract

The present work aimed to probe into the effect of long non-coding RNA (lncRNA) LINC00152 on gastric cancer (GC) cells proliferation by regulating *miR-193a-3p* and its target gene *MCL1*. Transfected si-LINC00152 was used to down-regulate LINC00152, and cells proliferation was measured by the cell counting kit-8 (CCK-8) assay. Cell apoptosis and cell cycle were analyzed by flow cytometry (FCM). Besides, we also detected the potential functional effects of differential expression of LINC00152 *in vivo* using nude mouse xenograft model. We overexpressed and downexpressed *miR-193a-3p* to study the *in vitro* effect of *miR-193a-3p* on GC cells proliferation and vitality. And *MCL1* was silenced by shRNA to investigate the effect of *MCL1* on proliferation of GC cells. In this research, LINC00152 was proven to have a higher expression level in GC tissues than in the adjacent normal tissues. GC cells proliferation was inhibited after LINC00152 was down-regulated. LINC00152 inhibited the expression of *miR-193a-3p*, which negatively regulated *MCL1*. In addition, GC cells proliferation was inhibited by cell transfection with shRNA-*MCL1*, and enhanced by transfection with *miR-193a-3p* mimics. Our study suggested that LINC00152 was overexpressed in GC tissues, and it down-regulated *miR-193a-3p* to enhance *MCL1* expression thereby promoting GC cells proliferation.

## Introduction

Amongst the most critical malignant neoplasms, gastric cancer (GC) is the second common leading cause of deaths relevant to cancer around the world [1]. Lamentably, early GC is difficult to diagnose because there are usually no specific symptoms, and remedial surgery is not an alternative for diagnosis [2]. To provide the foundation for molecular treatment approaches, it is necessary to have a clear understanding of molecular mechanisms behind the development and progression of GC [3].

Myeloid cell leukemia-1 (*MCL1*) is one of anti-apoptotic Bcl-2 family proteins with a short half-life period, and previous work has demonstrated that up-regulation of *MCL1* might inhibit apoptosis, chemoresistance, and cell cycle progression of tumor cells [4]. Moreover, some researchers have found that *MCL1* was overexpressed in a lot of human neoplasms. For example, the overexpression of *MCL1* regulates the cell growth in gastric neoplasms, being an obstacle of apoptotic signaling [5]. As a result, appropriately regulating the expression level of *MCL1* becomes a significant issue in GC treatment. The importance must be attached to tight regulation of *MCL1* expression in all kinds of biological processes related to gastric neoplasms [6].

In the last decade, advanced genomic analysis of genes expression has showed much more genetic transcription than hitherto expected. And the lion’s share of the genome was reported to be transcribed into non-coding RNAs (ncRNAs) [7]. Though ncRNAs were considered to be ‘noise’ at the beginning, piling up evidence has pointed out that ncRNAs, ranging from the small RNAs like miRNAs, siRNAs, piRNAs to the long ncRNAs (lncRNAs), serve as an important part in gene expression [1]. Recently, the new-found ncRNA, LINC00152, has been reported to be overexpressed in GC, which strongly indicates a relationship between LINC00152 and GC cells proliferation [8]. Furthermore, other studies have demonstrated that overexpression of LINC00152 was positively correlated with larger tumor volume, tumor invasion depth, higher TNM stage, and poorer livability [9]. Though LINC00152 was confirmed to play a critical role in the pathologic process of GC, the specific mechanism of LINC00152 involved and its target proteins or signaling pathway remained unknown [10].

MiRNAs are also a member of ncRNAs family with small volume (~20 nts), and miRNAs binding to the target mRNAs, regulating proteins expression by three approaches: controlling translation, increasing degradation of the target mRNA, and promoting translation at the post-transcriptional level [11]. MiRNAs, each has hundreds of target regions, can regulate the majority of genetic pathways and bind up to 30% of human genes [12]. It has been shown that down-regulation of *miR-193-3p* inhibits proliferation, migration, and chemotherapy resistance of tumor cells in GC through regulating *PTEN* gene [13]. Besides, previous work has confirmed that the transfection of *miR-193a-3p* decreases the expression of *MCL1*, and *MCL1* is a direct target of *miR-193a-3p* [6]. Furthermore, an interesting discovery is that LINC00152 works as a competing endogenous RNA (ceRNA) through sponging *miR-193a-3p* and shares the identical responsive elements of *miR-193a-3p* with some signaling pathway factor like erb-b2 receptor tyrosine kinase 4 (*ERBB4*) [14].

In this work, we worked over the relationship between LINC00152 expression and the cell multiplication of GC, and we verified both *in vivo* and *in vitro* that LINC00152 promoted gastric cells proliferation by regulating *miR-193a-3p* and its target gene *MCL1*.

## Experimental

### Cell culture and tissue samples

A total of 20 GC tissues and adjacent normal tissue samples were collected from patients undergoing curative cancer surgery at the Third Affiliated Hospital of Sun Yat-Sen University. Before the endoscopy examination, there was no chemotherapy or radiotherapy. After freshly freezing under liquid nitrogen, the specimens were stored at −80°C. Informed consent was obtained from all patients with experimental protocols receiving approval from the Ethics Committee of Third Affiliated Hospital of Sun Yat-Sen University. All patients were diagnosed with GC according to histological examination. The tissue samples were reviewed independently by three pathologists.

### Microarray

Based on the GPL570 platform and its correlated gene-expression profiling, GSE54129 was obtained from the Gene Expression Omnibus (GEO) database (http://www.ncbi.nlm.nih.gov/geo/). GSE54129 contained 111 cancer tissues and 21 normal adjacent tissues. Cut-off value for dysregulated lncRNAs was set at >two-fold change (FC) and *P*-value was <0.05.

### Cell culture

Four GC cell lines (MGC-803, AGS, SGC-7901, and BGC-823) along with the normal gastric epithelial cell line (GES-1) were purchased from the BeNa Culture Collection (BNCC, Shanghai, China). The cells were incubated in 90% RPMI-1640 medium (Gibco, #31800022) together with 10% FBS (Invitrogen, Carlsbad, CA, U.S.A.), and they were grown in adapt circumstances at 37°C with 5% CO_2_.

### RNA isolation and qRT-PCR

Expression levels of LINC00152, *miR-193a-3p*, and *MCL1* were determined by qRT-PCR. RNAs were extracted by TRIzol reagent (Invitrogen, Carlsbad, CA, U.S.A.) in light of the manufacturer’s protocol. The miRNA isolation was carried out from the total RNA using mirVana™ miRNA isolation kit (Ambion, Austin, TX). NanoDrop 2000 (Thermo Fisher Scientific Inc, Waltham, MA, U.S.A.) was used for quantitation, and afterward, RT-PCR was conducted by ReverTra Ace qPCR-RT Kit (Toyobo, Japan) as described in the protocol of the reagents. The obtained product was then analyzed by real-time quantitative PCR analysis using THUNDERBIRD SYBR® qPCR Mix (Toyobo, Japan). The relative expressions were normalized to GAPDH or U6. The relative expression results were computed by 2^−ΔΔ*C*^_T_. The primers (Sangon, Biotech, Shanghai, China) used are shown in Table 1.

**Table 1:** Primer sequences for qRT-PCR

Primer	Sequence (5′–3′)
GAPDH-F	5′-AAGGTGAAGGTCGGAGTCAA-3′
GAPDH-R	5′-AATGAAGGGGTCATTGATGG-3′
Linc00152-F-1	5′-GAAGGTGTCGGCAAGATC-3′
Linc00152-R-1	5′-TCGGTGTCTGTCATATTCG-3′
Linc00152-F-2	5′-CAGCACCTCTACCTGTTG-3′
Linc00152-R-2	5′-GGATTAAGACACATAGAGACTG-3′
si-linc00152	5′-AAUCUUUCAGCUGCAUUCCTT-3′
sh-linc00152	5′-CACCAATCTTTCAGCTGCATTCCTTCGAAAAGGAATGCAGCTGAAAGA-3′
MCL1-F	5′-GGGCAGGATTGTGACTCTCATT-3′
MCL1-R	5′-GATGCAGCTTTCTTGGTTTATGG-3′
*miR-193a-3p*-F	5′-ACTGGCCTACAAAGTCCCAGT-3′
*miR-193a-3p*-R	5′-GTGCAGGGTCCGAGGT-3′
U6-F	5′-CTTCGGCAGCACATATAC-3′
U6-R	5′-GAACGCTTCACGAATTTGC-3′

Abbreviations: F, Forward primer; R, reverse primer.

### RNAi

*MiR-193a-3p* mimics, *miR-193a-3p* inhibitor, and pcDNA3.1 plasmid vectors were purchased from GenePharma (Shanghai, China). The following groups were set: negative control (NC) group to be the group transfected with pcDNA3.1 empty plasmid vector, mimics group to be the group transfected with both *miR-193a-3p* mimics and pcDNA3.1 empty plasmid vector, inhibitor group to be the group transfected with both *miR-193a-3p* inhibitor and pcDNA3.1 empty plasmid vector, LINC00152 + mimics (mix) group to be the group transfected with *miR-193a-3p* mimics + pcDNA3.1-LINC00152. The sh-MCL1 and overexpressed MCL1 were transiently transfected to GC cells by Lipofectamine 2000. AGS and BGC-823 cell lines were incubated in six-well plates and transfected by Lipofectamine 2000 (Life Technologies Corporation, Gaithersburg, MD, U.S.A.) 24 h later. Cells were grown in adapt circumstances at 37°C with 5% CO_2_, and harvested at 48 h after transfection for further analysis. In animal study, AGS cells were stably transfected with sh-Ctrl or sh-linc00152 and then screened using 1 μg/ml puromycin (Beyotime, Shanghai, China) 48 h after the transfection. Stable clones were picked every 7 days of selection. Linc00152 expression levels were detected by qRT-PCR.

### Colony formation assay

Cells were digested with trypsin into single-cell suspensions at 48 h after transfection, and they were incubated in six-well plates containing 10 ml of prewarm RPMI-1640 medium. Cells were cultured in adapt circumstances at 37°C with 5% CO_2_. After 1 or 2 weeks, the cells were fixed with 4% paraformaldehyde for 15 min followed by staining with GIMSA (Seebio, Shanghai, China) for 15–30 min. Visible colonies were manually counted.

### Cell counting kit-8 assay

The ability of cells proliferation was assayed using cell counting kit-8 (CCK-8) (Biotech Well, Shanghai, China) in light of the manufacturer’s instructions. Logarithmically growing AGS and BGC-823 cells were taken out and digested with 0.25% (v/v) trypsin into single-cell suspensions, and the transfected cells were seeded in flat-bottom. Cells were cultured in adapt circumstances at 37°C with 5% CO_2_. CCK-8 was detected at 0, 24, 48, 72, and 96 h. The optical density (OD) was determined by a microplate reader at 450 nm.

### Flow cytometry assay

AGS and BGC-823 cells transfected were harvested 72 h after transfection by trypsinization. Supernatant of the mixture was discarded after centrifugation. The cells were fixed in 75% ethanol at 4°C for 4 h after washing with PBS. PI and RNase were used for staining. The cells for cell cycle analysis were then analyzed by FACS Calibur (BD Biosciences, San Jose, CA, U.S.A.). The data were analyzed using FACS Diva (BD, U.S.A.) software.

### Tumor formation assay in a nude mouse model

After stably transfecting and harvesting, washed AGS and BGC-823 cells were resuspended. Then suspended cells were injected into the left side of the posterior flank of each mouse subcutaneously, at an inoculation depth of 1 cm. Tumor growth was examined twice every week, and the volumes of tumors were computed by V = 0.5 × D × d^2^ , where V refers to volume; D means longitudinal diameter; and d stands for latitudinal diameter. At 4 weeks after injection, mice were mercifully killed, and then the subcutaneous growth of tumors was examined for later molecular analysis, immunohistochemistry, and Hematoxylin-Eosin (HE) staining assay.

### HE staining

The paraffin-embedded tumor tissues were cut into sections amongst the injection site and the growth and invasion of implanted tumor were observed by routine HE staining. All tissues were fixed for 1–3 s in 4% paraformaldehyde and then rinsed with running water, followed by 60-s Hematoxylin staining. After staining with Hematoxylin and rinsing with running water, the sections were soaked in hydrochloric acid solutions for 1–2 s, rinsed with running water, and then immersed in ammonia for 1–2 s. Then, the sections were rinsed with running water again, stained with Eosin solution for 30 s, followed by being rapidly dehydrated in graded ethanol, cleared in xylene, and mounted with neutral gum.

### Immunohistochemical analysis

Tumor sections were baked at 60°C for 2 h and then deparaffinized and rehydrated in xylene followed by graded ethanol. Antigen retrieval was performed by heating (100°C) in citrate buffer (10 mM, pH 6.0) for 25 min. Endogenous peroxidase was quenched with 3% hydrogen peroxide in methanol. Slides were blocked with goat serum for 15 min and then incubated at 4°C with primary antibody, anti-MCL1 (#ab32087, 1:100 dilution, Abcam, Cambridge, MA, U.S.A.) overnight. Sequentially, secondary antibody (Abcam, Cambridge, MA, U.S.A.) was applied at 4°C for 30–40 min. After washing with PBS, diaminobenzidine (DAB) was added for 10–20 min, followed by washing in water. Slides were counterstained for 30 s with Hematoxylin. At last, the sections were rapidly dehydrated, cleared in xylene, and mounted in neutral gum. The pathological sections were observed under the microscope.

### Western blotting

All the protein was extracted from cultured cells or tissues by RIPA (Beyotime, Shanghai, China) with protease inhibitor cocktail (Roche, Basel, Switzerland). The concentration of protein was measured by BCA Protein Assay Kit (Pierce, Rockford, IL, U.S.A.). Samples were loaded equally in lanes, resolved using SDS/PAGE (Beyotime, Nantong, China), and transferred on to a nitrocellulose membrane. The membranes were blocked at room temperature with 5% BSA for 1 h, and incubated overnight at 4°C with primary antibodies (anti-MCL1, #ab32087, 1:1000; anti-GAPDH, #ab181603, 1:10000, Abcam, Cambridge, MA, U.S.A.). Consecutively, the secondary antibodies (IgG-HRP, #ab7090, 1:2000, Abcam, Cambridge, MA, U.S.A.) were added and the protein was incubated for another 1.5 h at low temperature shaker. ECL Plus (Life Technology, Shanghai China) was used for protein visualization, and GAPDH was used for quantity normalization of the protein.

### Dual-luciferase reporter gene assay

The synthetic LINC00152 and LINC00152-mut sequences were inserted into the XbaI and FseI restriction sites with the pGL3 plasmid (Promega, Madison, WI). BGC-823 and AGS cells were transfected with pGL3-linc00152-WT or pGL3-linc00152-mut. Meanwhile, Lipofectamine 3000 transfection reagent (Life Technologies, U.S.A.) was used to co-transfect *miR-193a-3p* mimics or scrambles (mimics NC) into AGS or BGC-823 cells. The relative luciferase activities were normalized to *Renilla* luciferase activities by *Renilla* luciferase vector pRL-SV50 (Promega, Madison, WI). The luciferase activities were assessed at 48 h after transfection, using Dual-Luciferase Reporter Assay System (Promega, Madison, WI).

By the same method, *MCL1*-WT and *MCL1*-mut sequences were inserted into AGS and BGC-823 cells by the pGL3 plasmid, co-transfected with* miR-193a-3p* mimics or mimics NC. The luciferase activities were measured at 48 h after transfection.

### Statistical analysis

All the experiments in our study were performed in triplicate and repeated three times at least. One-way ANOVA was used to do multiple-group comparisons. Data were expressed in the format of mean ± S.D., and Student’s *t*test was performed to test the differences between two independent groups. All statistical analyses were presented with GraphPad Prism 6.0 software. *P*<0.05 was taken as statistically significant.

## Results

### LINC00152 was overexpressed in GC tissues

GSE54129, including 111 cancer tissues and 21 normal adjacent tissues, was acquired from the GEO database for microarray-based analysis. According to the microarray analysis, 126 lncRNAs were overexpressed and 82 lncRNAs were lowly expressed in the GC tissues, as shown in the volcano plot (Figure 1A) and the heat map (Figure 1B). Amongst them, LINC00152 expression in GC tissues was markedly increased, compared with adjacent normal tissues (*P*<0.01, Figure 1C and Supplementary Figure S1A). Besides, in AGS, SGC-7901, BGC-823, and MGC-803 cell lines, LINC00152 was obviously expressed at a higher level than in GES-1 cell line (Figure 1D and Supplementary Figure S1B).

**Figure 1:** LINC00152 was overexpressed in GC tissues and cell lines (**A**) Volcanic map showed the overall significantly differentially expressed lncRNAs in GC. (**B**) Heat map showed the differentially expressed lncRNA level between normal and tumor groups. (**C**) qRT-PCR showed that LINC00152 was overexpressed in GC tumor tissues (*n*=20), compared with normal (*n*=20). (**D**) LINC00152 was overexpressed in four different GC cell lines. GES-1 cell line was used as normal control. * represents *P*<0.05, ** represents *P*<0.01, compared with normal group.

### LINC00152 silencing inhibited GC cells proliferation

The knockdown efficiency of si-LINC00152 was evaluated in both AGS and BGC-823 cells (Figure 2A). The colony formation assay demonstrated that colonies were reduced remarkably in the si-LINC00152 group than in the si-NC group (*P*<0.05), indicating that LINC00152 silencing suppressed GC cells proliferation (Figure 2B), and CCK-8 assay detected cell viability in different time points also showed similar results (Figure 2C). Furthermore, the flow cytometry (FCM) assay was used to examine cell cycle progression, AGS and BGC-823 cells transfected with si-LINC00152 showed a cell cycle arrest at G_1_/G_0_ phase (*P*<0.01, Figure 2D).

**Figure 2:** LINC00152 regulated GC cells proliferation *in vitro* (**A**) The relative expression level of LINC00152 in AGC or BGC-823 cells transfected with si-NC or si-LINC00152. (**B**) The representative results of colony formation transfected with si-NC or si-LINC00152 in GC cells. (**C**) CCK-8 assays were performed to determine cells proliferation after transfection of siNC or si-LINC00152. (**D**) At 48 h after transfection, the cell cycle was analyzed by FCM. GC cells transfected with si-linc00152 were arrested in G_1_/G_0_ phase. * represents *P*<0.05, ** represents *P*<0.01, compared with NC group.

### Sh-linc00152 suppressed the tumor growth of GC cells *in vivo*

To validate the oncogenic role of LINC00152 in GC tumorigenesis, we constructed a xenograft mouse model. At 6th week after injection of stably transfecting sh-linc00152 or sh-Ctrl AGS cells, we found that knockdown of LINC00152 significantly decreased tumorigenesis. The tumors formed in the sh-linc00152 group of nude mice were notably smaller and lighter than those in the empty vector group (*P*<0.05, Figure 3A–C). qRT-PCR showed that LINC00152 expression was decreased in the sh-linc00152 tumor tissues, compared with the control group (*P*<0.05, Figure 3D). Furthermore, immunohistochemical (IHC) analysis indicated decreased MCL1 staining, and HE staining analysis reflected a lower rate of tumor proliferation, in tumor tissues with suppressed LINC00152 expression (Figure 3E). In short, our results revealed that sh-linc00152 inhibited the tumor growth of GC cells *in vivo*.

**Figure 3:** Sh-linc00152 inhibited tumor growth in the xenograft study (**A**) After 6-week incubation, the photograph of tumor size from differentially transfected groups. (**B**) The tumor growth curve. (**C**) The tumor weight was bigger and heavier in the sh-Ctrl group after 6 weeks. (**D**) The average expression of LINC00152 was lower in the sh-linc00152 group, compared with the control group. (**E**) HE staining and IHC staining illustrated that the expression of MCL1 was lower in the sh-linc00152 group. *, *P*<0.05, compared with sh-Ctrl group.

### The interaction between LINC00152/*miR-193a-3p* and *miR-193a-3p*/*MCL1*

TargetScan prediction output revealed that LINC00152 might contain a binding site for *miR-193a-3p* (Figure 4A), and* miR-193a-3p* might contain a binding site for *MCL1* (Figure 4C). To verify the above two predictions, pGL3-linc00152-wt (*MCL1*-wt) and pGL3-linc00152-mut (*MCL1*-mut) were constructed for dual-luciferase reporter assay. It was indicated that the target binding of linc00152-mut and *miR-193a-3p* was reduced (*P*<0.01, Figure 4B), and the target binding of *MCL1*-mut and *miR-193a-3p* was also reduced (*P*<0.01, Figure 4D), which was evidenced by significantly higher luciferase activity in mut groups compared with wt groups. Moreover, the overexpressed LINC00152 increased *MCL1* level, while the silenced LINC00152 increased *miR-193-3p* level. *MiR-193-3p* could also negatively regulate *MCL1* level (*P*<0.01, Figure 4E). In GC tumor tissues, the MCL1 expression level was positively correlated to linc00152 level (Figure 4F). Taken together, these data suggested that LINC00152 could directly interact with *miR-193a-3p*, and *miR-193a-3p* could directly interact with *MCL1* in GC cells.

**Figure 4:** LINC00152/*miR-193a-3p* or *miR-193a-3p*/*MCL1* had direct interaction (**A**) TargetScan prediction revealed that linc00152-wt could directly bind with *miR-193a-3p*. (**B**) Luciferase reporter gene assay verified that the binding intensity between linc00152-mut and *miR-193a-3p* was reduced. (**C**) TargetScan prediction revealed that *MCL1-*wt could directly bind with *miR-193a-3p*. (**D**) Luciferase reporter gene assay showed that the target binding of *MCL1*-mut and *miR-193a-3p* was reduced. (**E**) The regulation effect between linc00152/*miR-193-3p* or *miR-193-3p*/MCL1. (**F**) The expression relationship between linc00152 and MCL1 in tumor tissues. ** represents *P*<0.01, compared with NC groups.

### LINC00152 relieved cells proliferation inhibition induced by *miR-193a-3p*

To investigate the influence of *miR-193a-3p* on GC cells proliferation and the negative regulation effect of LINC00152 on *miR-193-3p*, we transfected mimics NC, *miR-193a-3p* mimics, *miR-193a-3p* inhibitor, *miR-193a-3p* mimics, and pcDNA3.1-LINC00152 into AGS and BGC-823 cells, respectively. The effectiveness of mimics and inhibitor transfection was confirmed by comparing with the control group. The lower expression of *miR-193a-3p* in the mix group compared with the mimics group validated that LINC00152 negatively regulated *miR-193a-3p* (*P*<0.01, Figure 5A). The colony formation assay revealed that the GC cells proliferation was suppressed after transfection with *miR-193a-3p* mimics, and the suppression was reversed by LINC00152 (*P*<0.01, Figure 5B). The CCK-8 assay showed that *miR-193a-3p* overexpression remarkably reduced cellular viability compared with control groups (*P*<0.05), while cellular viability of mix group (transfected with *miR-193a-3p* mimics and linc00152) was increased compared with the mimics group (Figure 5C). Besides, the FCM analysis indicated that *miR-193a-3p* overexpression significantly promoted the arrest of both cell lines in G_1_/G_0_ phase, with an obvious decrease in the number of S-phase cells (*P*<0.05). LINC00152 in the mix group reversed the cell reproduction arrest induced by *miR-129a-3p* (Figure 5D).

**Figure 5:** *MiR-193a-3p* inhibited GC cells proliferation *in vitro* (**A**) qRT-PCR revealed that the expression of *miR-193a-3p* was increased in the mimics group and decreased in the inhibitor group; linc00152 could reverse the increased *miR-193-3p* level of mimics group in AGS and BGC-823 cells, respectively. (**B**) The representative results of colony formation 1 week after the transfection. (**C**) In the CCK-8 assay, cell vitality was decreased in the mimics group and increased in the inhibitor group compared with the NC group, and cell vitality was increased in the mimics + linc00152 group compared with the mimics group. (**D**) FCM analysis indicated that *miR-193a-3p* overexpression significantly promoted the arrest of both the cell lines in G_1_/G_0_ phase, while mimics + linc00152 could reverse this effect. * represents *P*<0.05, ** represents *P*<0.01.

### *MCL1* promoted GC cells proliferation

Now that we have validated the direct interaction between *MCL1* and *miR-193a-3p*, we further confirmed the effect of *MCL1* on GC cells by transfecting NC, *MCL1*, sh-*MCL1* into AGS and BGC-823 cells, respectively. The expression level of *MCL1* was measured by both qRT-PCR and Western blot. The results revealed a decrease in *MCL1* expression in the sh-*MCL1* group, indicating the effectiveness of sh-*MCL1* transfection (*P*<0.05, Figure 6A,B). Overexpressed *MCL1* facilitated colony formation while sh-*MCL1* inhibited this tendency (*P*<0.05, Figure 6C). CCK-8 assay showed that *MCL1* enhanced viability and restricted apoptosis of GC cells (*P*<0.05, Figure 6D). Furthermore, the FCM analysis revealed that sh-*MCL1* significantly promoted the arrest of both cell lines in G_1_/G_0_ phase (*P*<0.01, Figure 6E). Collectively, the results suggested that *MCL1* positively affected GC cells proliferation.

**Figure 6:** *MCL1* promoted GC cells proliferation (**A**) The mRNA expression of *MCL1* was up-regulated in *MCL1* group, and down-regulated in sh-*MCL1* group. (**B**) Western blot revealed that the MCL1 protein expression was increased in *MCL1* group and decreased in the sh-*MCL1* group. (**C**) The representative results verified the promoted effects of *MCL1* on colony formation. (**D**) CCK8 assay indicated that cell vitality was increased in *MCL1* group, but decreased in the sh-*MCL1* group. (**E**) FCM analysis revealed that sh-*MCL1* significantly promoted the arrest of both two cell lines in G_1_/G_0_ phase. * represents *P*<0.05, ** represents *P*<0.01, compared with NC group.

### LINC00152 enhanced *MCL1* expression by down-regulating *miR-193a-3p*

To further investigate that whether *MCL1* expression was regulated by LINC00152 through *miR-193a-3p*, qRT-PCR, and Western blot were conducted to analyze the mRNA and protein expression of *MCL1* in *linc00152* or *miR-193a-3p* transfected cells. Amongst the five groups, the expression of *MCL1* was lowest in the *miR-193a-3p* mimics groups, while *MCL1* expression was enhanced in linc00152 and *miR-193a-3p* co-transfected groups compared with the mimics groups (*P*<0.05). Thus, the inhibition of *MCL1* given by *miR-193a-3p* was again confirmed by comparing the mix group to the LINC00152 group (*P*<0.01). Besides, cells in both the *miR-193a-3p* inhibitor group and LINC00152 group showed a higher *MCL1* expression than in the control group (Figure 7A). Similar results can be obtained from the Western blot assay, which showed the protein levels of *MCL1* in different transfection groups (Figure 7B). Furthermore, Kaplan–Meier survival analysis was used to examine the association between LINC00152/*MCL1* and GC patient prognosis. Moreover, patients expressing increased expression levels of LINC00152/*MCL1* had notably shorter survival time than those with low expression of LINC00152/*MCL1* (Figure 7C).

**Figure 7:** LINC00152 enhanced *MCL1* expression by down-regulating *miR-193a-3p* (**A**) The mRNA expression levels of *MCL1* when LINC00152 and miR-193a-3p were differentially expressed. (**B**) Expression of MCL1 protein when lLINC00152 and miR-193a-3p were differentially expressed. (**C**) When LINC00152 or *MCL1* was up-regulated, survival time was significantly reduced. * represents *P*<0.05, ** represents *P*<0.01.

## Discussion

Over the past 30 years, lncRNAs have proved to play an important role in various malignant tumors [9]. Amongst tens of thousands identified lncRNAs, increasing evidence has shown that LINC00152 was an oncogene involved in multiple cancers [15–17], and it was significantly overexpressed in various kinds of human cancer cell lines [18–22]. Studies revealed that silencing LINC00152 had marked effects to inhibit cells proliferation, invasion and migration, and enhance cell apoptosis [23]. Though LINC00152 was confirmed to be involved in cell cycle arrest and proliferation in GC [1], the detailed molecular mechanism of LINC00152 involved in GC tumor growth still needs further investigation. In the present work, we investigated the LINC00152 expression in GC tissues along with adjacent normal tissues in different cell lines. We finally came to a conclusion that LINC00152 was up-regulated in GC cell lines and tissues.

LINC00152 was identified to be one of the oncogenes that could be potential diagnostic/prognostic markers [24]. In this study, we observed remarkably higher expression level of LINC00152 in four GC cell lines (AGS, BGC-823, SGC-7901, and MGC-803) as well as human normal gastric epithelial cell line GES-1, consistent with the results given by Pang et al. [8]. Besides, we confirmed that knockdown of LINC00152 suppressed GC cells proliferation and the *in vivo* test verified that silencing LINC00152 decreased tumor size and weight.

Recently, Xia et al. [25] found that lncRNAs might play a crucial role in GC occurrence and development by interacting with miRNAs and participating in signaling pathways. Researchers have demonstrated that *miR-193a-3p* *serves* as a neoplasm suppressor in lung cancer [26,27] and colorectal cancer [28]. Besides, *miR-193a-3p* was identified as an antiproliferative miRNA inhibiting endothelial colony forming cells (ECFC)-derived cell proliferation [29]. In our study, a direct relationship between LINC00152 and *miR-193a-3p* was demonstrated. Furthermore, *miR-193a-3p* notably reduced proliferation and viability of GC cells, which was consistent with the results given by Pekow et al. [30]. That was to say, LINC00152 could relieve cells proliferation inhibition induced by *miR-193a-3p*.

*MCL1* has been proved to be overexpressed in GC tissues compared with normal gastric tissues [5] and was able to mediate the resistance to apoptosis in GC cells [31]. Previous studies revealed that *MCL1* was inversely correlated with the level of some miRNAs such as *miR-193b* [32] and *miR-125b* [3], and *MCL1* expression could induce epithelial–mesenchymal transition (EMT) via some signaling pathways, which subsequently stimulated the invasive and migratory capacity of human GC cells [4]. In the present study, we verified that *MCL1* silencing suppressed GC cells proliferation, and we further demonstrated that *miR-193a-3p* overexpression inhibited GC tumor growth by directly targetting at *MCL1*.

So far, we have demonstrated that up-regulation of LINC00152 suppressed *miR-193a-3p*, contributing to enhancement of *MCL1* expression and afterward, promoting proliferation of GC cells. In addition, we performed qRT-PCR and Western blot to further validate this assumption. Finally, we came to a conclusion that LINC00152 overexpression promoted GC cells proliferation by LINC00152/*miR-193a-3p*/*MCL1* pathway. The current study also had some unavoidable limitations; for example we conducted cell experiments mainly in AGS and BGC-823 GC cell lines, while the specific experiment results in other GC cell lines had missed. However, we believed that the tendency would be similar and this could be further investigated in the future. Collectively, our study showed LINC00152 might function as an oncogenic lncRNA to drive cancer development through LINC00152/*miR-193a-3p*/*MCL1* pathway and have great potential to become a promising biomarker and therapeutic target in GC.

## Conclusion

In summary, our study first proposed the LINC00152/*miR-193a-3p*/*MCL1* pathway involved in GC tumor development, and indicated the critical role of LINC00152 in GC cell proliferation. Our findings gave a clear understanding of how LINC00152 was involved in the tumor growth of GC cell proliferation, and it could serve as a potential target for therapy hereafter.

## Availability of data and materials

Please contact the authors for data requests.

## Consent to publish

Consent for publication was obtained from the participants.

## Supporting information

## Abbreviations

Bcl-2: B-cell lymphoma-2
CCK-8: cell counting kit-8
FCM: flow cytometry
GAPDH: Glyceraldehyde-3-phosphate dehydrogenase
GC: gastric cancer
GEO: Gene Expression Omnibus
HE: Hematoxylin-Eosin
HRP: Horseradish Peroxidase
IHC: immunohistochemical
lncRNA: long non-coding RNA
LINC00152: Long intergenic non-coding RNA Long intergenic no-coding RNA
*MCL1*: myeloid cell leukemia-1
NC: negative control
ncRNA: non-coding RNA
PI: Propidium Iodide
PTEN: Gene of phospjate and tension homology deleted on chromsome ten
qRT-PCR: Quantitative Real-time Polymerase Chain Reaction
RIPA: Radio Imminoprecipitation Assay
RPMI-1640: Roswell Park Memorial Istitute-1640
TNM: Tumor Node Metastasis
Xba1: Xanthomonas badirii 1
